The article "Long Noncoding RNA HLA Complex Group 18 Improves the Cell Proliferation of Myocardial Fibroblasts by Regulating the Hsa-microRNA-133a/Epidermal Growth Factor Receptor Axis" was retracted in 2023. Reasons: signs of a paper mill; suspected computer-generated content; unreliable results or conclusions; lack of ethics approval or compliance.

# Long Noncoding RNA HLA Complex Group 18 Improves the Cell Proliferation of Myocardial Fibroblasts by Regulating the Hsa-microRNA-133a/Epidermal Growth Factor Receptor Axis

**DOI:** 10.1155/2022/2668239

**Published:** 2022-07-31

**Authors:** Huoshun Shi, Lebo Sun, Dawei Zheng, Guodong Xu, Guofeng Shao

**Affiliations:** Department of Cardiothoracic Surgery, Lihuili Hospital, Ningbo 315048, Zhejiang Province, China

## Abstract

Hsa-microRNA (has-miR)-133a inactivates the extracellular signal-regulated kinase 1/2 (ERK1/2) pathway and suppresses the cell proliferation of myocardial fibroblasts by downregulation of the epidermal growth factor receptor (EGFR) expression. Bioinformatics analysis exhibits extended noncoding RNA HLA complex group 18 (lncRNA-HCG18) binds to hsa-miR-133a. The purpose of the current experiment is to explore whether lncRNA-HCG18 adsorbed hsa-miR-133a through sponging, resulting in decreased inhibition of hsa-miR-133a on EGFR and ultimately promoting the proliferation of myocardial fibroblasts. To verify and study the correlation and mechanism between lncRNA-HCG18, hsa-miR-133a, and their target genes. Firstly, after overexpression/silencing of lncRNA-HCG18 in myocardial fibroblasts, the level of hsa-miR-133a expression was evaluated by quantitative reverse transcription-polymerase chain reaction (RT-qPCR), and the EGFR, ERK1/2, and p-ERK1/2 expression levels were assessed by Western blotting to confirm that upregulation of EGFR and p-ERK1/2 protein levels by overexpression of lncRNA-HCG18, siRNA lncRNA-HCG18 (siHCG18) reduced the EGFR and p-ERK1/2 protein levels. Then, the luciferase reporter gene system was used to verify that lncRNA-HCG18 regulated EGFR expression by inhibiting the function of the hsa-miR-133a regulatory target gene. Then, a RAP assay was used to confirm that lncRNA-HCG18 interacted with hsa-miR-133a. Finally, the analysis of CCK-8 results indicated that the cell proliferation of myocardial fibroblasts was significantly reduced by siHCG18 while reversed by overexpression of lncRNA-HCG18. Thus, lncRNA-HCG18 inhibited cell viability of cardiac fibroblasts via the hsa-miR-133a/EGFR axis, which was regarded as a regulator of cell proliferation of cardiac fibroblasts in cardiovascular diseases.

## 1. Introduction

Long noncoding (lnc) RNA is an RNA transcript that is over 200 nucleotides long and has no open reading frame [1]. The roles of lncRNAs in regulating fibrosis are gradually being elucidated and have critical effects on various biological processes [2]. As epigenetic research progresses, the determination of lncRNAs can support new targets for the diagnosis, therapies, and prognosis prediction of myocardial infarction [3]. Reports have shown a significant correlation between cell proliferation of lncRNAs and myocardial infarction [4, 5]. Extended noncoding RNA HLA complex group 18 (lncRNA-HCG18) is a novel observed lncRNA that has been observed eccentrically in various diseases [6]. However, the mechanism of lncRNA-HCG18 regulating the cell proliferation of myocardial infarction cells remains unclear.

MicroRNAs (miRNAs) have been shown to play a role in cellular biological development, including cell proliferation, apoptosis, differentiation, and metabolism [7, 8]. MiRNAs play a central role in cardiac fibroblast metabolism [9]. MiRNAs maintain the metabolic balance of cardiac fibroblasts by regulating cell growth [10]. Hsa-miR-133a, a novel observed miRNA molecule, is closely associated with central nervous system (CNS) utilities and plays a regulatory effect on neural cell apoptosis and protection in the hippocampus [11]. However, it remains to be seen whether cardiac fibroblast growth is related to the expression abnormalities of hsa-miR-133a. Recent reports suggest that lncRNAs could play an essential role in gene regulation through miRNA adsorption [12, 13].

Studies have reported that the extracellular signal-regulated kinase 1/2 (ERK1/2) signaling pathway affects tumor cell proliferation mainly by regulating the progression of the tumor cell cycle [14, 15]. Currently, the expression, effect, and regulatory theories of the lncRNA-HCG18/hsa-miR-133a/EGFR axis in cardiac fibroblasts are limited. Hsa-miR-133a inhibits cardiac fibroblast growth by inactivating the ERK1/2 signaling pathway and down-regulating EGFR expression [16, 17]. Bioinformatics analysis shows that lncRNA-HCG18 could bind to hsa-miR-133a [6]. Therefore, we assumed that lncRNA-HCG18 adsorbed hsa-miR-133a through sponging, resulting in decreased inhibition of hsa-miR-133a on EGFR, promoting cell proliferation of myocardial fibroblasts. The main objective of the current experiment was to explore the theories of lncRNA-HCG18 in cell proliferation of myocardial fibroblasts and to determine the effect and interactions of the hsa-miR-133a/EGFR axis in the lncRNA-HCG18-mediated addition of myocardial infarction cells.

## 2. Reagents and Methods

### 2.1. Cell Incubation

Human cardiac fibroblasts (Ber004-J3) were obtained from Berginbio and preserved in Dulbecco Modified Eagle medium (DMEM, Hyclone; Cytival, USA) with penicillin (1%), streptomycin (1%, Gibco; Thermo Fisher Scientific, Inc., USA), and FBS (10%, Invitrogen; Thermo Fisher Scientific, Inc.). They were cultured in a humidified incubator (5% CO_2_, 37°C, 48 h).

### 2.2. Construction of High-Expression lncRNA-HCG18

The plasmid HKPCP-5 included the full-length cDNA of lncRNA-HCG18 and the vector pcDNA3.1-flag. After straightening the plasmid, PCR cloning was to place *BamHI* and *XhoI* restriction sites at the 5′- and 3′- ends of cDNA. Next, the PCR products were digested with the appropriate enzyme, reciprocated in *BamHI* and *XhoI*, cloned into pcDNA3.1-Flag induction/secreted expression vectors (Invitrogen, Thermo Fisher Scientific, Inc.), purified by gel, and dephosphorylated with shrimp alkaline phosphatase as recommended by the producer. Ligations were confirmed via enzyme digestion, and the nucleotide sequences were verified to be recombinant expression vectors with lncRNA-HCG18 nucleotide sequences and internal frame by deoxy seauencing.

### 2.3. Silencing lncRNA-HCG18 Expression

Three different concentrations of siRNA HCG18a (siHCG18a), siHCG18b, and siHCG18c were transfected using a mixture of siRNA (50 nm); scrambled was used as a control group (Thermo Fisher Scientific, Inc.). SiLENTFECT (BIO-Rad Laboratories, Hercules, CA, USA) transfection was performed according to vendor requirements. Cardiac fibroblasts were inoculated 8 h before transfection and transfected 2 days later.

### 2.4. Quantitative Reverse Transcription-Polymerase Chain Reaction (RT-qPCR)

The total RNAs were extracted from cardiac fibroblasts by a TRIzol reagent (Invitrogen, Thermo Fisher Scientific, Inc.). A nano-DROP 2000 spectrophotometer (Thermo Fisher Scientific, Inc.) was used to investigate the contents of the extracted RNAs. ReverTra Ace® qPCR RT Master Mix (BIO-Rad Laboratories) and gDNA Removal Kit (Toyo Textile, Osaka, Japan) were used to reversing RNA into complementary DNA. All surveys involve a minimum of three wells, each repeated three times. The LncRNA-HCG18 and hsa-miR-133a primers were developed according to the Sanguang Biotechnology Co., LTD. (Shanghai, China) and synthesized with U6 and glyceraldehyde 3-phosphate dehydrogenase (GAPDH), respectively (Table 1). Subsequently, RT-qPCR was investigated in 2 × RealStar Green Fast Mix kits (BIO-Rad, Laboratories). The 2^−ΔΔCt^ method was used in this experiment to calculate the folding change.

### 2.5. Western Blotting

The total proteins were isolated from cardiac fibroblasts that were western blotted using the monoclonal antibodies against EGFR (1 : 1, 000, Abcam, Cambridge, MA, USA), ERK1/2 (1 : 1, 000, Affinity, USA), and p-ERK1/2 (1 : 1, 000, Affinity). The loading control was served by GAPDH (1 : 1, 000, Sigma-Aldrich, USA). Cardiac fibroblasts were cultured at 25°C for 1 h with a horseradish peroxidase (HRP) labeled secondary antibody (1 : 1,000, Proteintech, Chicago, USA). Band density quantifications were investigated using an Odyssey Infrared Imaging System (LI-COR Biosciences, Lincoln, NE, USA).

### 2.6. Luciferase Reporter Assay

Mutants (MUT) EGFR-3 ′-UTR and wild-type (WT) EGFR-3′-UTR containing estimated binding sites for miR-133a were developed and inserted into a pmirGLO dual-luciferase reporter vector (Yeasen Biotechnology, Shanghai, China). Reporter vectors containing EGFR 3′-UTR MTT or WT and NC-mimics/hsa-miR-133a mimics were simultaneously transfected into cardiac fibroblasts and cultured at 45% confluence. The luciferase activity was measured by a dual-luciferase analysis system (Yeasen Biotechnology) after 48 h and standardized with carbamylated agents.

### 2.7. Analysis of RNA Immunoprecipitation (RIP)

The analysis of RIP was investigated to verify the interactions between lncRNA-HCG18 and hsa-miR-133a. Shortly, RIP was analyzed as described by the manufacturer using the EZMagna RIP RNA Binding Protein immunoprecipitation Kits prepared by Millipore (Millipore, Massachusetts, USA). RNA-lysis buffers dissolved different cell populations with protease inhibitors and RNase inhibitors. The cell lysates were then cultured with RIP buffers with magnetic beads containing Ago2 antibodies (Millipore). IgG was used as a negative control (input group). The coprecipitated RNA was isolated and measured by PCR after culturing at 4°C for 2 h.

### 2.8. CCK-8 Assay

The CCK-8 assay was used to analyze the cell viability. Cardiac fibroblasts were grown at 2–4 × 10^4^ cells/well in 96-well plates and incubated in an incubator (37°C, 5% CO_2_). The CCK-8 solution (0.5 mg/mL, Yeasen Biotechnology) was subsequently added to the medium to a final concentration and incubated for 4 h at 37°C. Optical density values (570 nm) were then measured.

### 2.9. Statistical Analysis

All data were analyzed by SPSS 22.0 software (IBM, Armonk, New York, USA). Mean ± standard deviation was used to measure the data. Analysis of Variance (ANOVA) and Tukey's postmortem tests analyzed comparisons among different groups. *P* < 0.05 was regarded to be statistically evident.

## 3. Results

### 3.1. Overexpression of lncRNA-HCG18 Analysis

PCR was designed using PCR with a method that included two specific restricted loci (*BamHI and XhoI*) to incorporate full-length lncRNA-HCG18 cDNA into the mammalian expression vector pcDNA3.1. The vector had 18 amino acid residues upstream of the lncRNA-HCG18 sequence as signal sequences and 23 amino acid residues downstream of lncRNA-HCG18, including V5 epitopes and His6 tags. Cardiac fibroblasts were transfected with a full-length, mature, secreted lncRNA-HCG18 gene vector. Recombinant lncRNA-HCG18 was excreted in a serum-free medium with a metallothionein promoter, purified by DEAE ion-exchange chromatography, and then purified by His label-friendly chromatography. In SDS-PAGE, lncRNA-HCG18 represented a single band with a distinct molecular weight, matching the size of the proteins according to the number of amino acids in lncRNA-HCG18 (Figure 1(a)). The determination of lncRNA-HCG18 was verified by analyzing western blotting (Figure 1(b)). Polyclonal antibodies were used to immunize chlorine with a unique peptide sequence from the amino and carbide terminus of lncRNA-HCG18 (Figures 1(c) and 1(d)).

### 3.2. Silencing lncRNA-HCG18 Expression

As exhibited in Figure 2, the level of lncRNA-HCG18 mRNA expression decreased in the siHCG18a and siHCG18c groups compared to the scrambled group (all *P* < 0.001). In the siHCG18b group, the lncRNA-HCG18 mRNA expression level was minimal. This finding indicated that transfection was effective in lncRNA-HCG18 silencing, so we used siHCG18c for further experiments.

### 3.3. The Regulation of Hsa-miR-133a Expressions in vecHCG18 and siHCG18 Treated-Cardiac Fibroblasts

The cardiac fibroblasts were analyzed by qRT-PCR to assess the induction of mRNA for hsa-miR-133a. Expressions of the mRNA for hsa-miR-133a were detected in the cardiac fibroblasts, as shown in Figure 3. Compared with the vec group, vecHCG18-treated cardiac fibroblasts showed apparent downregulation of mRNA expression of hsa-miR-133a (*P* < 0.001). The level of the hsa-miR-133a mRNA expression was significantly promoted by the treatment with siHCG18 compared with the scrambled group (*P* < 0.001).

### 3.4. The ERK1/2, p-ERK1/2, and EGFR Expression Levels in vecHCG18 and siHCG18 Treated-Cardiac Fibroblasts

The cardiac fibroblasts were analyzed by western blotting to assess protein induction for ERK1/2, p-ERK1/2, and EGFR. Expressions of the proteins for EGFR, ERK1/2, and p-ERK1/2 were detected in the cardiac fibroblasts, as shown in Figure 4. VecHCG18-treated cardiac fibroblasts showed apparent upregulation of EGFR and p-ERK1/2 protein expression levels (*P* < 0.001). VecHCG18 did not change the activation of ERK1/2 in the cardiac fibroblasts. siHCG18 reduced the EGFR and p-ERK1/2 protein expression levels (*P* < 0.001), while the ERK1/2 protein level exhibited no noticeable difference by treatment with siHCG18.

### 3.5. LncRNA-HCG18 Regulates EGFR Expression by Inhibiting Hsa-miR-133a-Regulated Target Gene Function

The results of the double-luciferase reporter gene test exhibited that the luciferase activity of EGFR-3′-UTR was apparently decreased (all *P* < 0.01) in the vec + hsa-miR-133a mimic, scrambled + hsa-miR-133a mimic, siHCG18 + mimic NC, and siHCG18 + hsa-miR-133a mimic groups as compared to that in the vec + mimic NC group. In contrast, the activity of pmirGLO exhibited no apparent influence on luciferase activity in these groups compared to that in the control group (*P* > 0.05, Figure 5). Additionally, in the vecHCG18 + mimic NC group, the luciferase activity of EGFR-3′-UTR was increased as compared to the vec + mimic NC group; also, in this group, the activity of pmirGLO exhibited no apparent influence on luciferase activity (*P* > 0.05, Figure 5). These data suggest that lncRNA-HCG18 regulates EGFR expression by inhibiting hsa-miR-133a-regulated target gene function.

### 3.6. RIP Analysis of the Interactions among lncRNA-HCG18 and Hsa-miR-133a

We used the RIP assay to verify the interactions among hsa-miR-133a and lncRNA-HCG18 in this study. The results of the RIP assay showed that has-miR-133a with lnc HCG18 was enriched in U6‐containing beads compared with the NC group (Figure 6). These data indicated that lncRNA-HCG18 interacted with hsa-miR-133a.

### 3.7. Effect of lncRNA-HCG18 on Cell Viability

The analysis of CCK-8 assays exhibited that after knockdown of lncRNA-HCG18 using siHCG18c, compared to the scrambled group, the cell proliferation was decreased, and the protective influences were suppressed (*P* < 0.05). As compared to the Vec group, higher cell proliferation was found in the vecHCG18 group (*P* < 0.05) (Figure 7). These data indicated that hsa-miR-133a inactivated the ERK1/2 signaling pathway by downregulating of the EGFR expression level and suppressing the cell proliferation of cardiac fibroblasts.

## 4. Discussion

LncRNAs regulate cell activity, including cell proliferation, apoptosis, differentiation, and metabolism [18]. Many studies have confirmed that lncRNAs play a critical effect in the occurrence, progression, development, and diagnosis of diseases [1, 4–6]. So far, many reports have explored the effect of lncRNAs in cardiovascular diseases [19, 20]. LncRNA-HCG18, a recently reported lncRNA, is eccentrically expressed in various conditions [6]. A bioinformatics analysis showed that lncRNA-HCG18 could bind to hsa-miR-133a [21]. Therefore, it was assumed that HCG18 adsorbed hsa-miR-133a through sponging, resulting in decreased inhibition of hsa-miR-133a on EGFR and ultimately promoting the proliferation of myocardial fibroblasts. In this study, the hsa-miR-133a level was evaluated by qRT-PCR after overexpression/silencing of lncRNA-HCG18 in myocardial fibroblasts. Then we found that vecHCG18-treated cardiac fibroblasts showed apparent downregulation of the mRNA level of hsa-miR-133a, while the mRNA level of hsa-miR-133a was significantly promoted by the treatment with siHCG18.

Studies have found that the ERK1/2 signaling pathway substantially affects the regulation of myocardial fibroblast proliferation and that this pathway affects cell proliferation mainly by regulating the progression of the cell cycle [14, 22, 23]. In addition, ERK1/2 is also closely related to cell invasion and metastasis [24, 25]. Activated ERK can activate protein-1 (AP-1) and nuclear transcription factor Kappa B (NF-*κ*B), promoting the matrix metalloproteinases-2/9 (MMP-2/9) activation, degrading the extracellular mechanism, allowing cells to penetrate the basement membrane, and promote the metastasis of myocardial fibroblasts [26, 27]. In the current study, vecHCG18-treated cardiac fibroblasts showed apparent upregulation of EGFR and p-ERK1/2 protein levels, and siHCG18 reduced the EGFR and p-ERK1/2 protein levels. At the same time, vecHCG18 or siHCG18 did not change the activation of ERK1/2 in the cardiac fibroblasts.

Reports have observed that the interactions among lncRNAs and miRNAs play a role in developing disease [28, 29]. More and more evidence found that miRNAs bind to the 3′-ends of significant transcription factors associated with cardiovascular disease [30]. MiRNAs can degrade target mRNAs or inhibit their translation [31]. Various miRNAs that regulate the course of cardiovascular disease have been reported [32]. For example, overexpression of miR-24 in cardiac fibroblasts and upregulation of miR-24 in cells inhibit the expression of genes related to cardiovascular disease and initiate the differentiation of fibroblasts into myofibroblasts [33]. A previous study has found that miR-214, miR-29, and miR-133a inhibit cardiovascular illness by suppressing the translational target gene expression of TGF*β*1, MMP2, and CTGF, respectively [34]. Studies have shown that hsa-miR-133a is significantly downregulated in HCC patients [35,36]. Our results found that hsa-miR-133a was the target gene of lncRNA-HCG18. In addition, overexpression of lncRNA-HCG18 decreased the expression level of hsa-miR-133a, while siHCG18 reversed the inhibitory effect of EGFR on hsa-miR-133a expression. Cell proliferation was reduced after knockdown of lncRNA-HCG18, and protective influences were impaired, while higher cell proliferation was found in the vecHCG18 group.

## 5. Conclusion

In conclusion, lncRNA-HCG18 inhibited the proliferation of cardiac fibroblasts through the hsa-miR-133a/EGFR axis, which provided a further elucidation of the theoretical basis for the molecular and biochemical mechanisms of the direct proliferation of cardiac fibroblasts in cardiovascular diseases.

## Figures and Tables

**Figure 1:** (a) The lncRNA-HCG18 expression was detected by PCR. (b) DNA electrophoresis map of lncRNA-HCG18 genes and their fragments identified by enzyme cutting after insertion into the expression vector. (c) LncRNA-HCG18 gene sequencing. (d) pcDNA3.1-flag-sequencing lncRNA-HCG18 cloning.

**Figure 2:** Silent expressions detection of lncRNA-HCG18 mRNA was evaluated by qRT-PCR. ^*∗∗∗*^*P* < 0.001.

**Figure 3:** The hsa-miR-133a mRNA expressions of vecHCG18 and siHCG18 treated-cardiac fibroblasts were detected by qRT-PCR. ^*∗∗∗*^*P* < 0.001.

**Figure 4:** The ERK1/2, p-ERK1/2, and EGFR protein levels of vecHCG18 and siHCG18 treated-cardiac fibroblasts were evaluated by western blot. ^*∗∗∗*^*P* < 0.001.

**Figure 5:** Luciferase reporter gene system confirms that lncRNA-HCG18 regulates EGFR expression by inhibiting miR-133a-regulated target gene function. ^*∗∗*^*P* < 0.01, ^*∗∗∗*^*P* < 0.001.

**Figure 6:** RIP experiments verify the interaction between lncRNA-HCG18 and hsa-miR-133a.

**Figure 7:** Cell viability was evaluated using the CCK-8 assay. ^*∗*^*P* < 0.05.

**Table 1:** Sequences for real-time PCR.

Gene	Sequence (5′-3′)
GAPDH	Forward AACGGATTTGGTCGTATTGGG
	Reverse CCTGGAAGATGGTGATGGGAT

LncRNA-HCG18	Forward GGGAGGAGAAAAAGTCCGGG
	Reverse GATAGGAGGAGTGAGTGCGC

Hsa-miR-133a	Forward TTTGGTCCCCTTCAACCAGCTG
	Reverse -

U6	Forward CTCGCTTCGGCAGCACA
	Reverse AACGCTTCACGAATTTGCGT

## Data Availability

The data used to support the findings of this study are included within the article.
